# Echoing Mechanism of Juvenile Delinquency Prevention and Occupational Therapy Education Guidance Based on Artificial Intelligence

**DOI:** 10.1155/2022/9115547

**Published:** 2022-09-29

**Authors:** Fang Hou

**Affiliations:** Research Centre of Applied Technology University, Huanghuai University, Zhumadian, 463000, China

## Abstract

In this paper, in-depth research and analysis of juvenile delinquency prevention and occupational therapy education guidance using artificial intelligence are conducted, and its response mechanism is designed in this way. Two crime type prediction algorithms based on time-crime type count vectorization and dense neural network and crime type prediction based on the fusion of dense neural network and long- and short-term memory neural network are proposed. The outputs of both are fed into a new neural network for training to achieve the fusion of the two neural networks. Among them, the use of the dense neural network can effectively fit the relationship between the constructed features and crime types. The behavioral manifestations and causes of the formation of deviant behavior in adolescents are discussed. They can only read numerical data, but there is a lot of information in the textual data that is closely related to the training effect. When experimenting, it is necessary to extract knowledge and build applications. The practical work with adolescents with deviant behaviors is again carried out from group work and casework, respectively, with problem diagnosis, needs assessment, and service plan development for specific clients, to carry out relevant practical service work. The causes of juvenile delinquency in the Internet culture are discussed in terms of the Internet environment, juvenile use of the Internet, Internet supervision, and crime prevention education, respectively. The fourth chapter focuses on the analysis of the prevention and control measures for juvenile delinquency in cyberculture. In response to the above-mentioned causes of juvenile delinquency in cyberculture, the prevention and control measures are discussed in four aspects, namely, strengthening the construction of cyberculture and building a healthy cyber environment, strengthening the capacity building of guiding juveniles to use cyber correctly, building a prevention and supervision system to promote the improvement of the legal system, and improving and innovating the crime prevention education in the cyber era.

## 1. Introduction

With the development of the economy and the influence of multidimensional values, weakening the mainstream values of society, adolescents also produce more significant behavioral deviations, although juvenile delinquency, in general, has moderated; they are prominent in the crime of minors but also the topic of public concern. Currently, juvenile delinquency is becoming increasingly complex in terms of violence, recurrence, and greed for profit, and although there are relatively more manifest characteristics, they all reflect a lack of self-control and social control [1]. As the future of the nation and the country depends on the youth, juvenile delinquency has become more complex as social transformation is accelerating. Traditional theories tend to analyze the causes of juvenile delinquency from a comprehensive perspective, suggesting that subject and extrasubjective factors jointly cause juvenile delinquency.

The study of juvenile crime early warning management promotes the integration of juvenile crime issues into the social early warning system and provides a new perspective and platform for juvenile crime prevention and reduction efforts. In terms of space, we will model the coordination and unification of several social management subsystems that are highly relevant to the development of youth education, such as comprehensive governance, public security, and political and legal affairs [2]. In terms of time, we will grasp the opportunity to prevent crime before it happens, take the initiative to carry out a targeted advance in advance, and transform the correction afterward into prevention and intervention beforehand; in terms of degree, we will establish a deep prevention and control pathway and through cooperation. The role of the implementation of juvenile crime prevention work improves the overall strategic deployment and improves the efficiency and effectiveness of the large system, to achieve a comprehensive approach to juvenile crime prevention and control work. Let the whole society pay attention to, care for, and care about juveniles, and take the initiative to carry out targeted early intervention to effectively prevent and control juvenile crime. Statistics on juvenile delinquency through the Youth Research Institute show that juvenile delinquency accounts for 70% of all delinquency cases nationwide. This frightening ratio highlights the urgency of the prevention of juvenile delinquency in China, and its data also shows that the age group of juvenile delinquency is controlled by the age group of 13 to 18 years old, and this age group accounts for 70% of all juvenile delinquency cases, and it is easy to see from the statistics and combing of the data that new crimes are committed in China every year [3]. The accuracy of the prediction results can reach more than 80% on the training subset and the test subset of the training set, but only a few percent accuracy on the test set. The reason is that this paper assumes that the experiment is ideally carried out in the state. At this point, the problem of juvenile delinquency is no longer a social concern, but an important issue that the country needs to control and prevent. How reduce and preventing juvenile delinquent activities is a common obligation of the state and the whole society.

Crime has certain spatial and temporal characteristics, so accurate prediction of the types of crimes that may occur in a certain spatial and temporal condition can enable public security organs to gain the initiative in dealing with delinquency cases, which is important for the improvement of the efficiency of public security organs. At the same time, only accurate prediction can play a positive role; the wrong prediction will not only mislead the public security organs' decision-making and deployment but also waste police resources and may cause significant social losses and personal casualties [4]. Therefore, countries all over the world attach great importance to crime intelligence forecasting, and some countries have set up special institutions for crime intelligence forecasting to organize experts and scholars for exploration. In the field of crime intelligence prediction, our scholars have also made some explorations. However, the research is still in the initial stage, and the research results are relatively scarce. On the one hand, some research directions are less explored, such as the prediction of case victims and the prediction of possible crime types under any spatial and temporal conditions; on the other hand, the energy of public security big data needs to be further activated by better prediction algorithms, the prediction accuracy needs to be further improved, and the stability of the generated prediction models needs to be further strengthened.

## 2. Related Works

Piquero et al. believe that interventions for aggressive adolescents can be carried out through joint discussions and role-playing and can achieve good service results [5]. Rackley et al. believe that social skills training and problem-solving training are necessary to reduce the risk of deviant behavior later in life because only after the youths have acquired the relevant social skills and learned how to solve problems, will they be able to cope with similar problems later in life [6]. The score is calculated by comparing with the real classification label, and the score at this time is an accurate assessment of the predictive ability of the model. This will reduce the likelihood of recurrence of deviant behavior and better adapt to the development of society. Molnar pointed out that in the prevention and intervention stage of adolescent deviant behavior, we need to carefully investigate and analyze the surrounding environment of adolescents and then cooperate with the family, school, community, and society to provide a good surrounding environment for adolescents [7].

Ziols et al. found that theft and fraud crimes are more likely to occur during the daytime, while robbery and snatching crimes mainly concentrated at night through statistical analysis of historical crime data [8]. Sun judged the crime situation and crime characteristics by conducting descriptive statistics on the number of criminal cases filed by public security organs nationwide and the number of criminal cases of theft and property fraud filed by public security organs nationwide from 2000 to 2014, thus predicting that the number of crimes will remain the same or decline slightly in 2015 [9]. Crime in the field of sociology can be regarded as a social transgression phenomenon with deep social structural roots. The study of student crime is mainly divided into crimes committed by secondary school students and college students according to different age stages and school types [10]. The percentage of teenagers who play games online is very high, and there are still many games on the market that are not suitable for teenagers. A variety of online games filled with brutal and bloody scenarios can deepen teenagers' recognition of violence and weaken instinctive morality. Teenagers have strong curiosity, are happy to imitate others' behavior, and are at a special age where they easily influenced and have more difficulty in distinguishing the boundary between the Internet and reality [11]. Online games containing violent elements do not only stimulate the senses of teenagers but also hinder their physical and mental development. Repeat crime refers to the same person having two or more criminal experiences. Repeat crime as a special crime phenomenon is analyzed separately from objective and subjective aspects: the objective sense indicates the depth of the criminal behavior of the perpetrator, and the subjective aspect can reflect the personal danger of the perpetrator [12]. At present, in many of the major cases and vicious cases in China, mostly repeat offenders, same in juvenile crime repeated criminal behavior is also more prominent.

People's understanding and view of crime are increasingly in-depth and comprehensive, and scholars at home and abroad have made some progress in the study of criminal intelligence prediction, realizing the leap from qualitative to quantitative, from artificial empirical methods to intelligent analysis methods, and from theoretical research to practical application, promoting the development of criminal intelligence prediction research in the direction of depth. However, it is undeniable that China's research started late, and relevant research results are still relatively scarce. There are more studies on crime trend prediction and crime quantity prediction and less on crime type and case victim prediction, more studies on prediction theory and less on the development of guided crime intelligence prediction models or auxiliary tools, more studies on descriptive analysis and less empirical studies based on valid data, and more studies on prediction using ordinary data mining algorithms. The research on the use of ordinary data mining algorithms for prediction is more frequent, and there are fewer attempts and innovations on advanced algorithms such as artificial neural networks; some scholars tend to pursue the complexity of the model in the research of establishing prediction models and believe that the hybrid model will have better prediction effect than the single model, but the prediction results not significantly improved in accuracy.

## 3. Analysis of Artificial Intelligence Method of Juvenile Delinquency Prevention and Occupational Therapy Education Guidance Echo Mechanism

### 3.1. Artificial Intelligence Crime Prediction Design

Compared to traditional programming methods, artificial neural networks do not require us to tell the computer how to solve the problem and break down the big problem into specific tasks at each step; it can learn automatically from the observed data and find the solution to the problem by itself. It is the feature of artificial neural networks to automatically learn features and process information that makes them play an important role in a growing number of industrial fields [13]. For example, it can be used in the medical field for disease identification; in the financial field for predictive analysis of stocks and marketable securities; in the communication field for recognition, denoising, compression, classification, and synthesis; in the commercial field for providing users with accurate advertising services; and in the chemical field for fault diagnosis, chemical engineering control, etc. Artificial neural network has a broad application prospect in many fields, and its characteristic of using a large amount of historical crime data more easily and more deeply to reduce data waste makes the artificial neural network more valuable for exploration in the field of public security.

A dense neural network is an artificial neural network composed of many layers of densely connected artificial neurons. According to the position of different layers, it can be divided into three kinds of layers: input layer, hidden layer, and output layer. Among them, the first layer is the input layer, the last layer is the output layer, the middle layers are all hidden layers, and the neurons between layers are fully connected. The network structure of the dense neural networks is the most typical and basic deep neural network structure. Therefore, a deep neural network (DNN) in the narrow sense refers to a dense neural network. If not specified, DNN in this paper refers to the dense deep neural network. However, the direct effect of school education on teenagers is 0.611, the direct effect of school education on legal education is 0.259, and the direct effect of playmate type is 0.226.

(1) $$\begin{array}{c} P_{A}=\frac{N_{f}}{N}-\frac{M_{f}}{M}. \end{array}$$

Firstly, the complexity of the network is low due to the small number of parameters. The first is the existence of a “local perceptual field”; each neuron of the convolutional kernel is no longer connected to all neurons in the previous layer, but only to a small number of neurons, which greatly reduces the parameter size of the neural network architecture compared with the fully connected form of traditional neural networks. Second, the model has good robustness. The weight sharing of the convolution kernel and the dimensionality reduction simplification of the downsampling layer make the feature extraction consider more mainly the relative position of a feature to other features without considering the specific position of each feature, so that even if the image is deformed by certain translation, scaling, distortion, and other deformation operations, the significant features can still be recognized and the “translation invariance” of the image can be realized. Therefore, compared with other neural networks, CNN is the primary choice for mining spatial correlation in data.

(2) $$\begin{array}{c} P_{a}=\frac{N_{f\_e}}{N_{E}}-\frac{M_{f_{e}}}{M_{E}}. \end{array}$$

Word vectorization is defined as an attempt to map words to vectors using a dictionary. In simple terms, word vectorization is the conversion of text into numbers, and the same text can be represented in different numerical forms. One reason a scholar performs vectorization is that computers are usually unable to effectively understand and process any valid output string or text [14]. And the local perception of neurons ensures that each region's own exclusive features are not affected by other regions; secondly, each convolution kernel shares the same weight and bias, instead of each connection having a different weight. Many machine learning algorithms and almost all deep learning networks cannot read strings or plain text in their raw form; they can only read numeric data, but there is a great deal of information in text-based data that is relevant to the training effect, from which knowledge must be extracted and applications built when experimenting. Therefore, text must be converted into numbers as input to perform any kind of work, such as classification and regression, in a generalized sense. Another reason of course is that neural networks are better at mining the hidden information between numbers during the learning process, as shown in Figure 1.

For example, firstly, the original data is divided into two parts, training set and test set, and the time-crime type count vectorization operation is performed on these two parts, respectively, which makes the training set and test set completely isolated; then, the training set is divided into two parts, training subset and validation subset, and training is performed on the training subset, and validation is performed on the validation subset, and then, suitable hyperparameters are selected. Finally, the model and hyperparameters obtained in the previous step are used for validation on the test set. Proper education to guide young people to understand what behaviors are not allowed by laws and regulations, and to lead by example in daily behaviors, is a key factor in whether the ward can act in accordance with legal norms. However, the experimental results show that, no matter how to debug, although the accuracy of the prediction results can reach more than 80% on both the training subset and the test subset of the training set, it can only reach a few percent accuracies on the test set, which is due to the assumption that the experiments are conducted under ideal conditions.

Before building the prediction model, 25% of the test set and 75% of the training set are randomly divided, and then, the features are normalized; i.e., the redundant parts of the data are eliminated so that the different features are comparable with each other. The algorithm to be used is then selected, and the modeling process can begin. The model-building process uses a 10-fold cross-validation technique in the training set, where all samples randomly divided into 10 groups, and then, one of the groups is selected as the validation set in turn, and the other nine groups are used as subtraining sets. The model is tested on the validation set using the model obtained in each subtraining set, and the model score is calculated.

After 10 training sessions, each set of samples is used 9 times as the subtraining set and 1 time as the validation set, and the scores obtained from the 10 cross-training sessions are averaged to obtain the final score of the model after the cross-validation technique. Finally, the prediction model obtained after cross-validation is tested on the test set to obtain the predicted classification results. The score is calculated by comparing it with the real classification labels, and at this point, the score is an accurate assessment of the model's predictive ability. After completing the prediction model, the importance of each predictor variable was also calculated; i.e., the features that played a significant role in the model were calculated.

Building the database is the most fundamental step in the exploration process of judicial big data and legal artificial intelligence [15]. If the whole exploration and construction process is compared to building a house, then the database is like the foundation, which needs to be as deep as possible to have a high house. This is dictated by the nature of big data analytics technology.

Both algorithms to improve accuracy and provide more learning objects for algorithms need the support of massive data, and even the quantity of data is much more important than the quality, as shown in Figure 2. Before the emergence of big data, people generally used sampling analysis to study information because they could not analyze the whole data. Due to the small sample size, it is necessary to ensure the accuracy of sampling for the precision of the results.

From the figure, the direct explanatory effect of the family economy on the fact of delinquency is 0, but the direct effect degree of school education for adolescents is 0.611, the direct effect of school education on legal education is 0.259, while the direct effect of playmate type is 0.226 and the direct effect of delinquency fact is 0.111. From the size of the labeled coefficients, legal education is the most important and direct kind of influence component, which acts directly on the fact of crime and has a weight of 0.392.

Because with the aggregation of massive data, inaccurate data will inevitably be mixed into the sample, but such inaccurate data is not unacceptable, because big data emphasizes more on the integrity and confusion of data, and the logic of big data analysis believes that no matter what kind of data is the reaction of the comprehensiveness of things, only through massive data can we further approach the truth [16]. With more data, the algorithm will improve the accuracy accordingly, to identify the inaccurate part of the data, which is why the foundation of big data and artificial intelligence construction lies in expanding the database.

### 3.2. Analysis of Juvenile Crime Prevention Occupational Therapy Education and Guidance Echoing Mechanism

Whether or not to pay attention to the comprehensive management of the juvenile growth environment will affect the education effect of juvenile legal consciousness, and whether juveniles have sounded their legal consciousness will ultimately affect the effect of national prevention and control of juvenile crime. In the commercial field, it can be used to provide users with accurate advertising services; in the chemical field, it can be used for fault diagnosis, chemical engineering control, etc. The growth environment of juvenile delinquency is complex, such as the failure of family function, the lack of legal education, and the degeneration of dating groups. Among them, as one of the elements of the growing environment, whether the direct caretakers and direct instructors of juveniles can improve their legal literacy, guide juveniles with appropriate education to know which behaviors are not allowed by laws and regulations, and set an example in their daily behavior is a key factor in whether the wards can act following the laws and regulations.

Because of the emulation characteristics of the youth group, their social differences are mainly reflected in two specific environments, namely, familiar playmates and social channels [17]. The Internet communication mode gradually replaces the traditional communication mode, and because the Internet information system in China has not been effectively regulated, it is full of some low-interest content that is harmful to the physical and mental health of adolescents. The model proposed to include the module of “social interaction,” including the types of playmates that adolescents often interact with and their use of the Internet, as shown in Figure 3.

At a certain stage of history, juvenile delinquency is inseparable from the development of society. Delinquency needs to be incorporated into social issues rather than simply being a problem of the criminal justice system. In this way, you can play different roles in the network and hide your real identity information and background information well. Therefore, crime prevention needs to be formed by the society with the corresponding capabilities and ideas and social control of juvenile delinquency, that is, based on social forces, to ensure that young people can recognize the mainstream social values and norms and follow them, making the process of effective maintenance of social order. The positive type uses praise, rewards, and other proactive methods to encourage those under control and ensure that some of their behaviors in line with social norms are maintained or reinforced. The negative type, on the other hand, uses punishment, demerits, criticism, and demotions to prohibit or limit the socially inappropriate behavior of the controlled person.

Since juvenile delinquency is socially deviant behavior and a serious one, it is an important disruptive factor that has a lasting impact on family relations and social stability, so social control is necessary for such behavior. Based on this need, a social control system to suppress juvenile delinquency was created.

This article starts from the background of practical research on the prevention of key juvenile delinquency, and with the premise of drawing on previous experience of the work of the Communist Youth League, it reorganizes and summarizes key juvenile delinquency and its related theories, trying to solve the problem of unclear and inaccurate positioning of the functions of the Communist Youth League in the process of preventing juvenile delinquency [18]. The article explores the effect of prevention of key juvenile delinquency using the method of case analysis, summarizes and analyzes the problems of participation in the prevention of key juvenile delinquency and its causes, and thus puts forward targeted opinions and suggestions for enhancing the prevention of key juvenile delinquency. We attempted to summarize and analyze the lessons learned from our predecessors and put forward a better improvement strategy in terms of establishing specialized institutions as well as improving the existing laws and regulations, expanding the participation area, and improving the organizational guarantee, as shown in Figure 4.

In the context of the process of the information age, the convenience, openness, and uncertainty of the Internet provide a breeding ground for juveniles to commit crimes secretly and conceal the consequences of crimes. Let the neural network better learn the correlation between crime time and crime type, to improve the accuracy of crime type prediction under this spatiotemporal condition. Youths involved in cybercrime can easily hide behind the computer screen by tapping the keyboard and mouse at their fingertips and can choose any time and space to operate without the constraints of time and space [19]. Internet subjects usually apply for accounts to carry out online activities, and criminals obtain multiple online accounts by certain means to play different roles in the network and hide their real identity information and background information well. Due to the imperfect regulation of the Internet, there are still many websites that do not require real-name authentication to apply for an account, or the audit of real-name authentication is not strict enough to screen out people with ulterior motives who use fake or untrue identity information to apply [20].

In real life, teenagers, as a special social group, are young and have a little social experience, so they do not often can express themselves freely, but the hidden nature of online culture allows teenagers to hide their social identities and gain more freedom of expression. When teenagers overly magnify this freedom, they will take advantage of the concealment feature of the Internet to follow their intentions and carry out relevant online activities without restriction, ignoring the restrictions of morality and law.

## 4. Analysis of the Results

### 4.1. Analysis of Artificial Intelligence Crime Prediction Results

In experiment 1, only the order of the data was simply considered, and all the data were sorted with the help of the new variable TIME, and then, the former was used as the training set, and the latter *X* data were used as the test set, and various values of *X* were taken to find that the best results were obtained when *X* = 1000, and the best accuracy was 0.035, and even the top-5 accuracy was only 0.126. The best results were still unsatisfactory. Although the experiment ensures that the past is used to predict the future and the prediction framework is more scientific and reasonable, the prediction result can only reach an accuracy of 0.035; i.e., the level of accuracy is the same as that of random guessing, so obviously, the role of artificial neural networks is not well played, and it can be said that experiment one is a failure.

The algorithm only mines the hidden correlation information between location and crime type in feature analysis, ignoring the depth value of temporal data. Therefore, this paper introduces time-crime type counting vectorized features to express the crime incidence at different time points and the crime rate of each crime type occurring at different time points through a new feature, so that the neural network can better learn the correlation between crime time and crime type, and thus improve the accuracy of crime type prediction under this spatiotemporal condition. To further distinguish the effect of special work on different receptors overall, the group level can also be divided. The new neural network structure is experimentally proven to perform better by replacing and adjusting the normalization function and regularization function and debugging the number of layers and neurons of the neural network.

First, in experiment 2, we introduced an upgraded version of the recurrent neural network LSTM with good performance in the field of time series prediction, and the training results were improved, with the accuracy of the test set reaching 0.101 and the top-5 accuracy reaching 0.394; second, in experiment 3, we established a DNN based on the confirmed optimal solution of the network structure and enhanced the data set by adding an operating system block. Both attempts resulted in significant improvements in the experimental results, as shown in Figure 5. The loss function is also chosen as the categorical cross-entropy, and the network is trained to improve the prediction effect by minimizing the distance between these two distributions. The Adam algorithm is chosen for the optimization function, which has a certain range of learning rates for each iteration of the parameters and does not cause the learning rate to become large because of a large gradient. This can lead to nonadaptive or biased behavior. Migrant children will inevitably have some negative emotions in the process of migration.

The values of the parameters are relatively stable and usually require no adjustment or only a little fine-tuning, which is simple to operate and computationally efficient, requires little memory, and has a relatively good working performance in many cases. The final experiment still uses accuracy as a measure of how well the model predicts.

It shows that the team has not changed her much, and in the future service, the differences of each team member need to be considered more carefully; the other seven team members feel that they are satisfied with the changes brought by the team. In this paper, we remedy this shortcoming by sorting the data with a new variable TIME and then dividing the training and testing sets in the order of time, so that the data used for testing must be located after the data used for training in the time order, which enables “predicting the future with the past” and makes the prediction more in line with the actual needs.

The logistic regression model was used to categorize the data and predict them in order of importance according to the importance coefficients of the variables. Learning stress dimension in stressful life events, social avoidance and distress dimension in social anxiety, social avoidance and distress dimension in social anxiety, positive affect, and family socioeconomic status, as shown in Figure 6. The importance of the interpersonal relationship dimension in stressful life events (0.530), the intimacy dimension in a teacher-student relationship (0.468), and the negative affect (0.426) were significantly greater than the rest of the influencing factors and were the main influencing factors of the problem behaviors of mobile children.

The importance of subjective family support ranked 3rd in the random forest, the importance of intimacy dimension in teacher-student relationship ranked 4th, and the conflict dimension in teacher-student relationship and peer status dimension in loneliness ranked 7th and 8th not represented in other models, indicating that the random forest approach can identify underappreciated variables in logistic regression and support vector machines. These variables are also likely to be important factors influencing the problem behaviors of mobile children and should also be considered. The 5th to 8th ranked importance variables in the logistic regression and support vector machine are family stress dimension in stressful life events, study stress dimension in stressful life events, fear of negative evaluation dimension in social anxiety, and social avoidance and distress dimension in social anxiety, respectively, and the 9th and 10th ranked variables only differ in order. The rankings were generally similar.

General stress theory suggests that individuals can develop negative emotions due to interpersonal tensions and thus can exhibit nonadaptive or deviant behaviors. Mobile children will inevitably develop negative emotions such as sadness, tension, and anxiety during their mobility. The short-term presence of negative emotions can help mobile children adapt to their new environment faster, while long-term negative emotions can affect the psychological health of mobile children.

### 4.2. Results of Occupational Therapy Education Guidance Response Mechanism

To verify whether the group activities achieved the expected goal, a satisfaction survey was conducted especially for the group members. The first is whether the group members are satisfied with the content of the group activities; the second is whether the group members are satisfied with the overall process of the group; the third is whether the group members are satisfied with the social workers and other staff; the fourth is whether the group members are satisfied with the help they received from the group, and the fifth is whether the group members are satisfied with the changes brought to them by the group. A five-point scale was used, with 5 being very satisfied, 4 being relatively satisfied, 3 being generally satisfied, 2 being relatively dissatisfied, and 1 being very dissatisfied. The rating scale of group members' satisfaction with group activities is shown in Table 1.

From Table 1, we can see that the satisfaction scores of group members with the content of group activities are all 4 or 5, which means that the group members are satisfied with the content of group activities; the satisfaction scores of group members with the overall process of the group are all 4 or 5, which also shows that the overall process of the group is recognized by the group members; the satisfaction scores of group members with the social worker and staff are all 5. At present, juvenile delinquency is becoming increasingly complex and has the characteristics of violence, repetition, and greed for profit. Although there are relatively many characteristics, they all reflect the lack of self-control and social control. The satisfaction ratings of the group members for the social workers and staff members are all 5, which means that the whole process of the group has been recognized and supported by the group members. The group members all felt that the group had brought them help and they were satisfied with this help because they all rated this help as 4 or 5; one group member gave only 3 points for the changes brought to her by the group, which means that the changes brought to her by the group were not very big, and it is necessary to consider the differences of each group member more carefully in the future service; the other seven group members felt that they were satisfied with the changes brought to them by the group. The remaining seven members felt that they were satisfied with the changes brought by the group. Therefore, overall, the group members were satisfied with the group service activities, and the group service was recognized by the group members.

Combining the contents of the variables attributed to different factors, this paper names the factors as key quantitative factors, including the implementation of financial guarantee, inclusion in the comprehensive governance assessment, the construction of the rights protection team, and publicity and education, which are indicators corresponding to the 1st level of juvenile crime early warning management work. In addition, quantitative indicators should be artificially added to the reflected content, which originates from the fact that the scientific comprehensive evaluation must rely on quantifiable quantitative indicators, and the key quantitative indicators cannot be separated from the accuracy and detail of basic data. However, we need to clearly recognize that the factors that control crime have not changed significantly. This control model has not been able to fully integrate extrasubjective and subject-based factors and has not been able to effectively connect the relationship between youth, natural, and social factors. The indicators that need to be included include crime rate, major vicious criminal cases, and other indicators, which are important quantitative measurement bases for evaluating the effectiveness of juvenile crime early warning work. The former focuses on the quantitative level of crime, while the latter reflects the characteristics and patterns of crime. To further distinguish the effects of special efforts on different receptors in the long term, group levels can also be divided. In the horizontal cross-sectional evaluation, homogeneous indicators of the same year and different regions are compared; in the vertical time-series evaluation, the progress and effectiveness of the glimpse management work of local departments are assessed in a specific period, as shown in Figure 7.

The Internet is a product of the times with outstanding instrumental properties, and young people carry out crimes related to the Internet, and the Internet should indeed be regulated in terms of influencing crime, but it can also play its positive significance in crime prevention education. According to statistics on juvenile delinquency by the Youth Research Association, juvenile delinquency accounts for 70% of the national crime cases. In the context of the prevalence of digital information exchange mode, it is quite feasible to make use of the east wind of the flourishing network to give full play to the instrumental value that the network has. As a new information and cultural communication medium, the information conveyed by the Internet has a natural attraction to teenagers compared with that conveyed by traditional platforms. Therefore, the publicity and education information on crime prevention can be more effectively received and accepted by the youth group by releasing it in the most frequently contacted network platform of youth, thus significantly improving the effectiveness of the publicity and education work on crime prevention for youth. In addition, a way to connect online networks and offline practice can be used to attract more youths to actively participate in crime prevention education activities.

## 5. Conclusion

There are more complex causes of juvenile delinquency and relatively more theories. Traditional prevention theories mostly analyze them to extrasubjective and subjective factors, but these analyses have not been able to effectively address the interface between the two factors. After a detailed discussion, this paper suggests that the key cause of juvenile delinquency is the lack of good self-control and self-concept in socialization and interaction with society. In this paper, we introduce the time-offense type counting vectorization feature, which expresses the incidence of crime at different time points and the incidence of each crime type at different time points through a new feature, so that the neural network can better learn the correlation between crime time and crime type and thus improve the accuracy of crime type prediction under this spatial and temporal condition. It is an important issue that a country needs to control and prevent. How to reduce and prevent juvenile delinquency activities is the common obligation of the state and the whole society. A more scientific and perfect early warning model of juvenile crime is initially constructed. On this basis, the evaluation method of juvenile crime early warning management is studied, and a multilevel hierarchical analysis model of juvenile crime early warning management, a multilevel comprehensive evaluation model of juvenile crime early warning management, and a gray system comprehensive evaluation model of juvenile crime early warning management are established. Finally, the mechanism and strategy of juvenile crime early warning management are studied and described. The stage measures of juvenile crime early warning are elaborated in three-time dimensions: prewarning, midwarning, and postwarning; meanwhile, specific strategies for juvenile crime are proposed in four methodological dimensions: family protection, school protection, social protection, and judicial protection.

## Figures and Tables

**Figure 1:** Artificial intelligence crime prediction model.

**Figure 2:** Four-factor path diagram of two exogenous variables of juvenile delinquency.

**Figure 3:** Juvenile crime prevention education and guidance response mechanism.

**Figure 4:** The means and tools of serious violent crimes committed by minors.

**Figure 5:** Experimental results of a crime database.

**Figure 6:** Characteristics of the top ten ranked by average importance in the regression algorithm.

**Figure 7:** Indicator mono-element evaluation results.

**Table 1:** Group members' satisfaction with group activities.

Name	Type A	Type B	Type C
A	4	3	4
B	6	4	6
C	3	3	6
D	5	4	5
E	4	3	3
F	4	4	3
G	6	5	5
H	4	4	3

## Data Availability

The data used to support the findings of this study are available from the corresponding author upon request.
